The article "Effect of 1 + N Extended Nursing Service on Functional Recovery of Colostomy Patients" was retracted in 2023. Reasons: signs of a paper mill; suspected computer-generated content; unreliable results or conclusions; concerns about the data.

# Effect of 1 + N Extended Nursing Service on Functional Recovery of Colostomy Patients

**DOI:** 10.1155/2022/2645528

**Published:** 2022-08-29

**Authors:** Chunlan Feng, Caixia Lv, Xia Zhang, Yumei Guo, Xiaojun Li

**Affiliations:** ^1^Department of Nursing, Wuwei Cancer Hospital, Wuwei 733000, Gansu, China; ^2^Department of Nursing, Heavy Ion Center of Wuwei Cancer Hospital, Wuwei 733000, Gansu, China

## Abstract

To many hospitals' management as well as to patients, the nursing service is one of the most important aspects. Many diseases like sugar, blood pressure, urine passage, and gas are a little bit dangerous to handle by patients themselves. The earlier stage models are unable to give good services to patients; therefore, an advanced JHE: Effect of 1 + N extended nursing service is necessary to crossover the above limitations. Colostomy and colorectal cancers are very dangerous syndromes thus, disease monitoring is so difficult. In this research work, an extended JHE: Effect of 1 + N extended nursing service modeling is discussed with experimental modeling. Apart from conventional nursing care provided by the observation group, it was given online training as well as service providing. Self-efficacy and self-care competence were assessed in both groups 6 months after the discharge. Quality of life and mental health were also assessed. Besides, their dimensional and total self-care ability scores, and the observation group's self-efficacy ratings were substantially higher than those of the control group (*P* 0.05) after the intervention. It was observed that the intervention group's 6-month adjustment to the stoma was statistically more favorable than the control group's (*P* 0.001), and only the intervention group showed a significantly major change (*P* 0.001) between their two evaluations. This proposed methodology can improve the accuracy rate by 93.23%, and succussive treatment rate of 92.14% had been attained.

## 1. Introduction

Approximately 700,000 people worldwide die each year from Colorectal cancer (CRC; also known as bowel cancer), colon cancer, or rectal cancer, which is the fourth most frequent kind of cancer overall. In the US, CRC 1 claimed the lives of 50,260 individuals in 2017. When it comes to colorectal cancer, males are more likely than women to be affected. After lung and prostate cancer, colon malignancies (CRC) in males ranked third in 2012 in Indonesia, whereas in women, it was second. A colostomy is the best option if CRC affects the rectum and the gastrointestinal system as shown in Figure 1. Colostomy frequently causes patients to feel weird and difficult to care for themselves, and this may lead to a reduction in their lifespan quality, which includes physical, psychological, social, and spiritual components. As many as 63% of individuals reported peristomal skin issues in the first 21 to 40 days after a colostomy. A stoma may also lead to complications such as varicose veins and peristomal hernias. It is impossible to prevent the complication of peristomal hernias, which have a substantial influence on the patient's quality of life (QoL) and comfort. About 70.00% of individuals with stomas have difficulties, and the risk of issues continues throughout their lifetimes. Patients' capacity for self-care, including managing their colostomy, is critically dependent on the work of nurses. Since getting used to living with a colostomy takes time, patients who have had colostomy surgery may find it difficult to return home.

The article "Effect of 1 + N Extended Nursing Service on Functional Recovery of Colostomy Patients" was retracted in 2023. Reasons: signs of a paper mill; suspected computer-generated content; unreliable results or conclusions; concerns about the data.

Enterostomal Therapy (ET) nurses may help patients' quality of life (QoL) after a colostomy by educating nurses and offering follow-up programs. Referring to the expertise and experience of the ET nurses, the requirement for follow-up is essential. ET nurses may use a variety of educational intervention methods to help patients improve their psychosocial and self-management abilities. Discussion in a chronic care group on colostomy self-care curriculum to increase HRQOL and self-management for patients' QoL and cost savings may be achieved via experience-sharing group education programs, involving stoma care and social activities, as well as organized educational programs. As a result, in the first year after a colostomy, ET nurses and systematic follow-up play a critical role in improving quality of life and reducing the severity of peristomal skin diseases (PSCs).

Technology, especially the telephone, may be used for follow-up. Patients may better control their chronic conditions by employing technology, such as mobile phones. Nurse-led follow-up calls are acceptable, appropriate, and successful when they are used in conjunction with telephone service. Nurses should make phone calls to patients who have returned for follow-up appointments because they are a confident, compelling, and rapid means of communication that encourages open dialogue about patient issues and allows nurses to give the appropriate answers. But nurses require solid communication skills in order to communicate with patients and help them improve the quality of their own self-care. In order to share information, give health education and guidance on the treatment of symptoms, reassure patients, and provide high-quality services, a telephone follow-up is a great option. The postdischarge TFU service provided by nurses is acceptable. In addition to improving the patient's quality of life, nurses may give emotional support, contentment, safety, and knowledge about treatment options via their follow-up care of cancer patients. Telephone follow-up is an alternative to regular hospital follow-up by tracking the adverse special effects of therapy and giving malignant cells patients with educational materials.

The article "Effect of 1 + N Extended Nursing Service on Functional Recovery of Colostomy Patients" was retracted in 2023. Reasons: signs of a paper mill; suspected computer-generated content; unreliable results or conclusions; concerns about the data.

The follow-up using smartphones has evolved as a way to provide excellent service lasting 10–15 minutes while simultaneously reducing hospital visits. Even regular phone and home visits, as well as in-hospital consultations with ET nurses, may address a range of problems, but the optimum follow-up method has yet to be determined. With a colostomy for 3 months, intensive TFU decreased complications, enhanced standard of living, and boosted satisfaction levels among patients.

TFU is beneficial to individuals with a permanent colostomy in several trials. They were only small-scale qualitative investigations and not randomized, and they failed to reveal the duration, kind, and amount of outcomes and assessments on TFU further. As a result, further research into the effects of TFU on people with permanent colostomies is required. People who have permanent colostomies were the focus of this study, which attempted to characterize and evaluate the impact of TFU on them methodically. RCT review articles are ideal for establishing a link between an intervention and its observed effects.

The contribution of this research work is an extended JHE: Effect of 1 + N extended nursing service modeling is discussed with experimental modeling. Aside from conventional nursing care provided by the observation group and it was given online training as well as service providing.

## 2. Literature Survey

Wabl et al. suggested that a severe traumatic brain injury (sTBI), DFR is often described but a few research has examined DFR after severe cerebrovascular brain damage (sCBI). A DFR lasting more than 1 to 3 months or 6 to 12 months was found in a similar percentage of those with sTBI as in those who had had a major stroke, suggesting that there is no discernible difference between the two [1].

Portinari et al. suggested that the goal of this study was to investigate the impact on postoperative recovery and cost-effectiveness of an Italian academic center's colorectal enhanced recovery program. It is practical, successful, safe, and cost-effective to use colorectal enhanced recovery programs for functional recovery and to shorten the length of hospital stays. Protocol adherence is necessary for both patient satisfaction and reduced nurse strain [2].

Colwell et al. assessed the expenses and incidence of peristomal skin complications (PSCs) associated with the use of ceramide-infused ostomy skin barriers (OSBs) and control OSBs. To be clear, these findings were based on exploratory research, rather than statistical analysis. With the application of a ceramide-infused barrier, the expenditures were considerably decreased and patient satisfaction was much increased [3].

The article "Effect of 1 + N Extended Nursing Service on Functional Recovery of Colostomy Patients" was retracted in 2023. Reasons: signs of a paper mill; suspected computer-generated content; unreliable results or conclusions; concerns about the data.

Peters et al. suggested that recovery from colorectal resection is made more difficult by ileus and anastomotic leaks that occur postoperatively. Patients were randomly assigned (1 : 1) to receive either continuous lipid-enriched enteral tube feeding from three hours before surgery until 6 hours afterward (intervention) or no perioperative nutrition using online randomization software with block sizes of six and stratified by location (colonic or rectal) and surgery type (laparoscopic or open) (control). Preoperative lipid-enriched enteral diet shows no benefit over conventional treatment in terms of postoperative complications in patients having elective CRC surgery [4].

Platt examined many aspects of SCI care in the ICU such as inpatient rehabilitation and outpatient rehabilitation settings from the patient's and the stakeholders' perspectives. This research yields a complete list of prospective prospects. Existing, developing, and future solutions to SCI patients' demands were taken into consideration while rating each high-potential opportunity. Patients' quality of life might be improved by using a wireless closed-loop neuromuscular electrical stimulation system [5].

Montroni et al. proposed that a patient-centered approach to treating rectal cancer in the elderly is essential in order to get the best possible outcomes. Patients in this age group are equally as important in terms of functional recovery and patient-reported outcomes as cancer-specific outcomes. The best available evidence led to the establishment of these and supplementary recommendations for the treatment of elderly people with rectal cancer [6].

Rojanasarot assessed the effect on avoidable healthcare usage of a postdischarge ostomy support program in addition to nurse-led ostomy care. These people were asked a series of questions about ostomy surgical features, readmissions, and emergency room visits within or after 1 month of discharge (including explanations for avoidable occurrences), as well as their degree of access to health care. Postdischarge ostomy support program enrollment seems to be a good strategy for cutting down on unnecessary medical expenses [7].

In Forsmo et al., the primary goal of this randomized controlled experiment was to examine the effect of additional preoperative counseling on postoperative recovery in otherwise indistinguishable patients. To minimize the duration of hospital stay, we found that preoperative counseling helps patients adhere to all aspects of postoperative improved recovery. https://ClinicalTrials.gov was notified about this investigation [8].

The article "Effect of 1 + N Extended Nursing Service on Functional Recovery of Colostomy Patients" was retracted in 2023. Reasons: signs of a paper mill; suspected computer-generated content; unreliable results or conclusions; concerns about the data.

In a controlled experiment by Wang et al., self-efficacy was substantially greater among patients in the intervention group than those in the control group at 01-, 03-, and 6-month follow-up (all *P* 0.05). At 1, 3, and 6 months following discharge, the incidence of stoma complications in the intervention group decreased. The results showed that stoma patients who get follow-up therapy through a mobile app may enhance their psychosocial adjustment, self-efficacy rating, and other outcomes [9].

In Xu et al., colostomy patients with rectal cancer were the focus of their study, which sought to examine the impact of thorough postdischarge care on their clinical outcomes. In this regard, the treatment deserves widespread use and promotion in clinical practice [10].

Jin et al. suggested that patients with stomas fared better under continuing care than under standard care in terms of health outcomes and satisfaction. We came up with a variety of proposals for implementing an integrated continuing care program [11].

Protocol compliance, surgical stress, and functional recovery will be examined in this study's primary focus. The results of a multivariate analysis were used to determine the influence of independent variables on functional recovery. Colorectal surgery patients who adhere to the ERAS procedure are less stressed and recover more quickly [12].

Elderly patients are commonly mistreated because of their age or their level of infirmity, or a combination of the two. Before surgery, it is critical to assess frailty and identify areas for intervention and optimization. Functional rehabilitation and quality of life are other important considerations that should be included in a patient's treatment plan from the outset. Geriatric patients may and should get individual treatment. Throughout a patient's life, geriatricians should be engaged in the care of the elderly [13].

SAS and SDS scores increased considerably in both groups after the intervention, with the observation group having significantly higher SAS and SDS scores than the control group (*P* 0.05). 6 months after the procedure, there were considerably fewer complications in the observation group than in the control group (*P* 0.05). Using an online training method that emphasizes self-care and self-efficacy may help patients with permanent enterostomies improve their quality of life and psychological well-being, while also reducing the likelihood of complications following discharge. [14].

The article "Effect of 1 + N Extended Nursing Service on Functional Recovery of Colostomy Patients" was retracted in 2023. Reasons: signs of a paper mill; suspected computer-generated content; unreliable results or conclusions; concerns about the data.

In the cohort of Saur et al., functional recovery and quality of life should be assessed. Cancer patients have a difficult time communicating, which becomes more difficult as they become older. In the care of elderly people, communication is essential. Research should concentrate on improving communication and assessing the quality of life and recovery indicators in the future [15].

The purpose of the study by Sheng and Mengxiao was to assess the well-being of the participants. An enterostomy may have a detrimental effect on patients' quality of life, according to studies. To help nurses better understand how stomas affect patients' life, this research yielded a variety of results [16].

Black and Notter the importance of quality of life (QoL) has grown over the last three decades, and it is now considered a critical assessment. To better assist stoma patients, health care providers should do more to help them adjust to living with a stoma and throughout their whole lives [17].

Mohamed et al. suggested that the burden of ostomy management for colorectal cancer patients was exacerbated by changes in food and nutrition. Both patients and caregivers agreed that seeking out counseling and other types of social support may help with the emotional adjustment to living with an ostomy. Ostomy patients' and caregivers' outcomes may be improved by creating and implementing an appropriate supportive care plan [18].

In Song et al., a self-management program for patients with recurrent rectal cancer who had colostomies was provided to them, and after its implementation, the occurrence of stomal and peristomal disorders was evaluated. As a result, data were collected from 43 participants in the intervention group and 42 participants in the control group.

Patients in the control group received typical post-hospital care, including stoma care instructions and twice-monthly telephone follow-ups for three months after discharge from the hospital. Those in the investigational group got a self-management program through a multimedia messaging app, which was accessible for 6 weeks following discharge, in addition to regular treatment. As a secondary result, we looked at the frequency of stomal and peristomal problems in addition to the primary outcome of self-efficacy and self-management capacity. Peristomal problems were shown to be less common in those in the intervention group, while stomal complications were not affected by the treatment. Peristomal problems were reduced in patients with colostomies who participated in a multimedia messaging app-based self-care programmer, according to the results of the study [19, 20].

In most of the existing systems, the evaluation is done with less number of patients, the hospital stay is not minimized in the existing system and the rate of recovery is also lower. To overcome these limitations, this article is proposed.

The article "Effect of 1 + N Extended Nursing Service on Functional Recovery of Colostomy Patients" was retracted in 2023. Reasons: signs of a paper mill; suspected computer-generated content; unreliable results or conclusions; concerns about the data.

## 3. Methodology

There is a significant incidence and mortality rate for rectal cancer in the US, making it one of the most common cancerous tumors of the gastrointestinal process. There has been a progressive decrease in the average age of rectal cancer incidence in recent years, but the incidence rate has been steadily rising. Early clinical indications of the condition are mild. Most patients with rectal cancer must have surgical resection as the foundation of their therapy, and they must wear a colostomy bag permanently [2]. Because of this, patients' quality of life and health are adversely affected by colostomy, which modifies their original manner of defecation and renders them unable of controlling it themselves. Because of this, nurses are increasingly concerned about the care of patients with rectal cancer who have to endure long-term colostomy removal [3]. In-patient treatment may be extended and maintained with continuous nursing, resulting in a better quality of life for the patient after they are discharged [4]. Over the previous several years, Chinese academics have made great progress in the field of clinical nursing by using the continuous nursing paradigm. Using online training and ongoing nursing care, this study evaluated the influence of network training on health-related quality of life and self-efficacy in patients with a permanent colostomy who had had surgery for rectal cancer as shown in Figure 1. You can see the results in Figure 2.

### 3.1. Clinical Materials

There were 119 individuals with rectal cancer who were hospitalized for permanent colostomy tubes inserted in the period from January 2018 to December 2019. The control group included 57 patients hospitalized between January 2018 and December 2018, whereas the observation group included 62 individuals admitted between January 2019 and December 2019. It was decided to proceed with this investigation by the Hospital Ethics Committee.

### 3.2. Criteria That Include and Exclude

#### 3.2.1. Inclusive Criteria

Patient eligibility was based on four main factors, all of which had to be met: (1) they had colorectal cancer diagnosed according to Chinese Medical Association cancer science branch diagnostic criteria; (2) they had no recurrence or metastasis of the tumor; (3) they were aged 20–70 years; and (4) they signed informed consent freely.

#### 3.2.2. Exclusive Criteria

To qualify, patients must meet the following criteria: (1) a problem with communication, understanding, or reading; (2) a history of radiation, chemotherapy, or immunotherapy; and (3) an abnormality in a crucial organ.

The article "Effect of 1 + N Extended Nursing Service on Functional Recovery of Colostomy Patients" was retracted in 2023. Reasons: signs of a paper mill; suspected computer-generated content; unreliable results or conclusions; concerns about the data.

## 4. Methodology

Frequent follow-up treatment was provided to the control group, which included health education at discharge and notification of regular follow-up hospital visits.

Continuous nursing care for the observation group was provided by defining the content as follows: Four nurses, one chief nurse, and one supervising nurse were part of the team that was organized to provide continuous nursing care. The team personnel got training from the physician and the head nurse in order to understand the study goals and the duties and responsibilities assigned to each member of the team. Knowledge of rectal cancer colostomy, adversely caused emotions of patients, and variables impacting life quality after colostomy were among the topics covered in the course. Patient files were established at discharge, and individualized medical nursing programs, including psychology, daily diet, disease reexamination, and exercise were implemented by the physician and nursing staff. Patients' knowledge of health education was strengthened, including self-care for patients, colostomy knowledge, and prevention and management of complications. New approaches and products were also introduced to help patients better integrate into their daily routines and strengthen their confidence in beating the condition. Instant Messaging groups like We Chat and QQ groups were created for patients and family members to post their daily self-care diaries on these platforms. A patient's medical history was entered into a nursing journal, and the staff kept track of any unusual occurrences, notifying patients to return to the hospital as soon as possible. Nurses answered patients' inquiries at predetermined times each week and performed video conversations once a month to monitor patients' emotional states and connect with them in a timely way. Patients were reminded by the medical personnel of the necessity of arriving on time for their appointments and were kept up to date on the latest developments in their treatment for rectal cancer and colostomy. In response to the patients' unpleasant responses, the nursing program was promptly altered in accordance with the self-care diary. A public account must be established. Health information, such as health recommendations, hilarious jokes, inspiring videos, and so on, were published in the official account of the department to assist ease the patients' stress and reconcile the connection between the nurse and patient.

### 4.1. The Study of Indices

1. For the pre- and post-treatment (6 months after discharge) assessment of self-efficacy in the two groups, researchers used the General Self-Efficacy Scale (GSES). Based on the work of a German psychologist, the Schwarzer Scale is very reliable and valid. Scale consisted of a total of ten things, and each item had four levels, each with a score ranging from 1 to 4, with the highest level being absolutely erroneous. The higher the score, the more confident one felt in general.
2. Before and after therapy (6 months after discharge), patients' self-care abilities were assessed using the Self-care Ability Scale (ESCA). Four categories were included in the ESCA Scale, each having a total score of 172: nursing concept, nursing knowledge, nursing responsibility, and nursing abilities. Patients with higher scores had a greater capacity for self-care.
3. Before and after the intervention, we utilized the MOS 36-Item Short Form Health Survey (SF-36) to assess life quality (6 months after discharge). Among the eight components of Sf-36 are the following: physiological function, role-physical pain, social function, mental health, role-emotional well-being, vitality, and overall well-being. Each dimension was given a score ranging from 0 to 100. Better exam scores were linked to a better quality of life.
4. It was determined that patients' mental health was assessed using the SAS and the SRS before and six months after the intervention (6 months after discharge) (SDS). More than a hundred points on each scale indicated more worry or despair.
5. Complications that occurred within 6 months after release from the hospital in the two groups were documented.

The article "Effect of 1 + N Extended Nursing Service on Functional Recovery of Colostomy Patients" was retracted in 2023. Reasons: signs of a paper mill; suspected computer-generated content; unreliable results or conclusions; concerns about the data.

### 4.2. A Study of the Data

Analysis of the data was done using SPSS22.0 and Excel. Data from both enumeration (*t*-test) as well as measurement (chi-squared) were examined using these two tests. a *P* value of 0.05 was deemed statistically significant.

## 5. Results and Discussion

### 5.1. Material Comparisons in the Medical Field

Table 1 shows that there were no significant variations in clinical materials between groups of individuals (*q* > 0.05).

### 5.2. Between Pre- and Post-Intervention Assessments of Self-Sfficacy

Preintervention variations in self-efficacy ratings across groups were not statistically significant (*P* > 0.05). Afterward, the interference, both collections' self-efficacy ratings, was considerably more advanced than before (*P* 0.05), and the directory of the observation group after the intervention was clearly greater than that of the switch cluster (*P* 0.05), as shown in Table 2 and Figure 3.

### 5.3. Patients' Abilities to Care for Themselves Before and After Treatment

Table 3 shows that self-care ability was substantially greater in the involvement collection than in the control group (*P* 0.05). However, the indices of the observation group after intervention were significantly higher than those of the control group shown in Tables 2 and 3.

The article "Effect of 1 + N Extended Nursing Service on Functional Recovery of Colostomy Patients" was retracted in 2023. Reasons: signs of a paper mill; suspected computer-generated content; unreliable results or conclusions; concerns about the data.

### 5.4. A Comparison of the Two Groups of Patients' Quality of Life Before and After Treatment

See Tables 4 and 5 for more details. The SF-36 scores of both groups rose significantly after intervention, and the observation group seemed to have higher SF-36 scores after intervention than the control group (*P* 0.05).

### 5.5. Pre- and Post-Intervention Psychological Assessments of the Two Groups

As demonstrated in Table 5; Figures 2 and 3, both groups had increased SAS and SDS grades postintervention, and the observation group had significantly higher SAS and SDS scores than the control group (*P* 0.05).

As shown in Figures 4 and 5., when compared to the control group, a *P* 0.05 was found for the difference between the two groups.

### 5.6. Complication Rates in the Two Groups are Compared

As shown in Tables 7 and 8, the observation group's 6-month complication rate was significantly lower than the control group's (*P* 0.05).

As shown in Table 9, a prevalent intestinal malignancy is rectal cancer. As people's eating habits and lifestyles evolve, so do the incidence, disability, and death rates for those suffering from rectal cancer, all of which are on the rise. Postoperative permanent colostomy and laparoscopic surgical excision of tumor tissue are common clinical procedures used to relieve patients' suffering. It's tough to adjust to a colostomy, which may lead to bad feelings and a worse quality of life for the patient, but it's worth it in the long run. As a result, appropriate nursing interventions are required for patients with rectal cancer who have had a permanent colostomy.

Nursing care offers prompt, accurate, and focused counseling to patients via follow-up visits, illness reexamination, patient fellowship, and new communication methods. Postoperative quality of life is improved by ongoing nursing care that helps patients move from the hospital to their families in a more efficient manner, which has a positive impact on society. In this study, a network education model for continuous nursing care is developed by combining a traditional on-site model with a cutting-edge online platform.

Patients' physical function, as well as their mental and emotional emotions, are all targets of modern medical therapy. Self-efficacy is a term used to describe a person's perception of their own abilities, judgments, and beliefs about their ability to do a task to a given level. Patients' self-efficacy, self-confidence, and motivation to make their own decisions and take control of their own treatment are all emphasized in this paper. Lifelong colon ostomy is an ongoing condition, and patients' mood, quality of life, subjective well-being, etc., are all factors in treatment success. Patients in both groups had significantly higher self-efficacy scores after intervention than before, and those in the observation group had significantly higher self-efficacy scores than the control group; after intervention, patient scores in both groups had significantly higher preintervention scores, and scores the observation. Through the use of online platforms and continuous nurse involvement, patients and their families were able to engage in the self-care process, which improved their self-efficacy and capacity to care for themselves, similar to previous researchers' findings. Medical personnel may assist patients in establishing self-care files, document patient self-care behavior, and play a role in reminding patients of the need of excellent care throughout continuous nursing care. Both patients and healthcare providers should be able to see that their actions are being monitored and rewarded in real time, which may be accomplished by using videos, social media platforms, and regular hospital visits to urge patients to take better care of themselves.

The article "Effect of 1 + N Extended Nursing Service on Functional Recovery of Colostomy Patients" was retracted in 2023. Reasons: signs of a paper mill; suspected computer-generated content; unreliable results or conclusions; concerns about the data.

Preintervention assessments of SF-36 considerably improved in both groups after the intervention, with the observation group reporting higher scores than those of their counterparts. In research, postdischarge health education and life counseling may assist patients to obtain more relevant information, developing healthy behaviors, and improving their quality of life after hospital discharge. While patients in the observation group saw a significant improvement in their quality of life, patients in the control group saw only a modest improvement, which may be linked to their failure to receive timely help following discharge and the medical staff's inability to implement an effective intervention, according to the findings of this study.

Subjects in the observation group showed considerably greater improvements in their psychological well-being than those in the control group after effective continuous nursing care. This may have something to do with increasing patients' self-efficacy and capacity to care for themselves. Patients who practiced good self-care were able to have greater control over their illness, which in turn helped them feel better mentally. Regular communication between medical professionals and patients may help patients' psychological well-being, boost their self-esteem, and enhance the nurse-patient bond throughout the self-care process after release from the hospital. Complication rates were also lower in the observation group than in the control group, which suggests that patients' capacity to care for themselves has improved as a result of a long-term caring intervention.

The article "Effect of 1 + N Extended Nursing Service on Functional Recovery of Colostomy Patients" was retracted in 2023. Reasons: signs of a paper mill; suspected computer-generated content; unreliable results or conclusions; concerns about the data.

The small sample size and short postoperative observation duration hampered this study's ability to conclude. Patients' postoperative living circumstances will be studied for a longer period of time thanks to an improved nursing model, a larger sample, and increased observation duration in the follow-up study.

With the use of online training-based continuous nursing care, patients who have been diagnosed with rectal cancer and who have a permanent colostomy may enhance their quality of life and lower their risk of problems after discharge.

To examine the impact of a stoma nursing care programmer on the individual's ability to adapt to an ostomy in their body. A controlled experiment with a control group was found that in the first and sixth-month following discharge from the hospital, patients with stoma were separated into two groups (the intervention group and the control group). In order to gather data, we used the Elimination Ostomy Adjustment Scale. The results of the *t*-tests were analyzed. It was observed that the intervention group's 6-month adjustment to the stoma was statistically more favorable than the control group's (*P* 0.001), and that only the intervention group showed a significantly major change (*P* 0.001) between their two evaluations. These findings show an impact on stoma adjustment, and the intervention programmer continues to be beneficial six months following hospital release. Positive effects on ostomy adjustment have been shown with the use of systematic treatments carried out by an ostomy care professional nurse.

## 6. Conclusion

Many hospital administrators and patients value the nursing staff highly. Some disorders, such as diabetes, high blood pressure, urinary tract infections, and gas, might be risky for individuals to treat on their own. To overcome the limitations of prior models, an enhanced JHE: Effect of 1 + N extended nursing service model is required. Colitis and colon cancer are very deadly, making disease monitoring difficult. With experimental modeling, an extended JHE: Effect of 1 + N extended nursing service model is examined in this study. Other than typical nursing care, the group received online training and service provision in addition to observation. Six months following discharge, both groups were tested for self-efficacy and self-care competency. Mental well-being and quality of life were also taken into consideration. After the intervention, the observation group's self-efficacy ratings were significantly higher than those of the control group (*P* 0.05), in addition to their dimensional and total self-care ability scores. It was observed that the intervention group's 6-month adjustment to the stoma was statistically more favorable than the control group's (*P* 0.001), and that only the intervention group showed a significantly major change (*P* 0.001) between their two evaluations. This proposed methodology can improve the accuracy rate by 93.23%, succussive treatment rate of 92.14% had been attained. Patients' postoperative living circumstances will be studied for a longer period of time thanks to an improved nursing model, a larger sample, and increased observation duration will proceed in future studies.

The article "Effect of 1 + N Extended Nursing Service on Functional Recovery of Colostomy Patients" was retracted in 2023. Reasons: signs of a paper mill; suspected computer-generated content; unreliable results or conclusions; concerns about the data.

## Figures and Tables

**Figure 1:** Colorectal cancer (CRC).

**Figure 2:** Representation of colostomy bag.

**Figure 3:** Assessment of the two groups' efficacy before and after the intervention.

**Figure 4:** Preintervention and postintervention comparison of SAS scores. When compared to the control group, a *P* 0.05 was found for the difference between the two groups. As shown in Table 6.

**Figure 5:** The SDS scores of the two groups before and after the intervention are compared.

**Table 1:** Clinical materials comparison between two groups.

Medical data	Identification module	Controlling factor	*S*/*y*^2^	*Q*
Male	037	031	00.339	00.560
Female	025	026		
Age	045.82 ± 7.02	046.18 ± 8.12	00.259	00.796
Married	048	041	00.475	00.491
Single	014	016		
Jr. high school or below	017	015	00.018	00.829
High school and above	045	042		
Private treatment	021	023	00.535	00.465
By social security or public expense	041	034		

**Table 2:** Self-efficiency score.

	Before intervention	After intervention
Observation group	19	23
Control group	19	21

**Table 3:** Self-efficiency comparison between two groups before and after intervention ($\bar{x}\pm s$).

Cluster	Count of cases	Past interposition	Later interposition	*t*	*P*
Opinion set	63	19.83 ± 1.62	22.17 ± 2.01	13.713	0.001
Switch cluster	58	19.21 ± 1.72	20.06 ± 1.93	6.513	0.002
*T*	—	0.621	6.621	—	—
*P*	—	0.515	0.0007	—	—

**Table 4:** Self-efficiency comparison between two groups before and after the intervention.

Metrics	Identification model				Control model			
	Count of cases	Past interposition	*t*	*P*	Count of cases	Past interposition	*t*	*P*
Self-caring models	21.07 ± 2.71	26.75 ± 3.22^a^	8.744	≤0.001	21.75 ± 3.22	25.03±	4.335	≤0.001
0.000 knowledge of self-care	28.97 ± 3.74	39.10 ± 5.70^a^	11.654	≤0.001	29.19 ± 5.300	33.66 ± 5.33	5.330	≤0.001
Responsibility of self-care	22.37 ± 2.36	28.29 ± 3.12^a^	13.500	≤0.001	25.39 ± 2.80	25.34 ± 2.30	6.281	≤0.001
Self-care skills	28.06 ± 4.24	42.01 ± 7.23^a^	12.990	≤0.001	33.56 ± 6.33	33.55 ± 6.30	5.098	≤0.001
Total score	98.93 ± 15.28	140.74 ± 21.33^a^	12.096	≤0.001	99.78117.29 ± 17.99	117.29 ± 17.99	5.521	≤0.001

The article "Effect of 1 + N Extended Nursing Service on Functional Recovery of Colostomy Patients" was retracted in 2023. Reasons: signs of a paper mill; suspected computer-generated content; unreliable results or conclusions; concerns about the data.

**Table 5:** Quality of life comparison among 2 groups.

Metrics	Identification model				Control model			
	Count of cases	Past inter position	*t*	Count of cases	Past inter position	After intervention	Count of cases	Past inter position
Physical functioning	58.55 ± 6.22	72.83 ± 5.89${}^{\underline{\text{a}}}$	13.133	0.000	0.75 ± 3.22	65.03 ± 92.00	4.789	0.000
Physical role	52.14 ± 4.20	26.75 ± 3.22^a^	11.315	0.000	50.19 ± 5.300	56.66 ± 5.33	6.587	0.000
Bodily pain	45.12 ± 3.58	39.10 ± 5.70^a^	18.148	0.000	44.39 ± 2.80	55.34 ± 2.30	9.587	0.000
Social functioning	46.88 ± 6.20	28.29 ± 3.12^a^	11.322	0.000	46.56 ± 6.33	61.55 ± 6.30	4.687	0.000
Mental health	53.62 ± 6.20	42.01 ± 7.23^a^	14.352	0.000	52.254 ± 17.99	63.29 ± 17.99	10.478	0.000
Emotional role	55.62 ± 6.99	140.74 ± 21.33^a^	12.235	0.000	55.75 ± 3.22	45.03 ± 5.145	7.315	0.000
Validity	55.20 ± 6.99	26.75 ± 3.22^a^	12.740	0.000	39.19 ± 5.300	56.66 ± 5.33	6.350	0.000
General health	40.20 ± 4.75	39.10 ± 5.70^a^	14.025	0.000	44.39 ± 2.80	57.34 ± 2.30	5.614	0.000

**Table 6:** SAS score analysis.

	Before intervention	After intervention
Observation group	60	45
Control group	60	54

**Table 7:** SDS analysis.

	Before intervention	After intervention
Observation group	59	43
Control group	60	51

**Table 8:** Physical states comparison between two groups.

Group	No. of cases	SASDS	SDSDS
Identification model	Past interposition	61.88 ± 6.33	60.21 ± 6.55
	Earlier interposition	49.88 ± 5.45	47.99 ± 4.79
	*T*	11.446	11.698
	*P*	0.00	0.000

Control model	Past interposition	61.22 ± 7.55	60.55 ± 7.23
	Earlier interposition	55.21 ± 6.23	52.44 ± 4.33
	*T*	5.247	7.422
	*P*	0.000	0.000

**Table 9:** Complication rates among 2 groups.

Group	No. of elements	Colostomy injury	Colostomy attack	Colostomy refutation	Contact	Total
Identification model	63	0 1 (0.000)	01 (0.000)	2 (1.62)	3 (3.23)	3 (4.85)
Control model	58	02 (3.57)	02 (1.75)	3 (3.52)	5 (7.03)	9 (14.78)
*T*	—	—	—	—	—	3.928
*P*	—	—	—	—	—	0.048

## Data Availability

No data were used to support this study.
